# Changes in Pre- and Postsurgery for Drug Resistant Epilepsy: Cognition and Sleep

This article has been retracted.

**DOI:** 10.1155/2022/9971780

**Published:** 2022-01-21

**Authors:** Lihong Li, Jun Lu, Yan Xu, Yuanyuan Zhao

**Affiliations:** ^1^Department of Acupuncture, The Second Affiliated Hospital of Zhejiang Chinese Medical University, Xinhua Hospital of Zhejiang Province, Hangzhou 310000, China; ^2^The Basic Medical College, Zhejiang Chinese Medical University, Hangzhou 310053, China; ^3^Department of Neurosurgery, Zhejiang Provincial People's Hospital, People's Hospital of Hangzhou Medical College, Hangzhou 310014, China

## Abstract

**Background:**

Most patients with drug-resistant epilepsy (DRE) have cognitive impairment and sleep disturbance. There was a significant correlation between sleep disorders and cognitive dysfunction. This study performed surgical treatment on patients with DRE and observed seizures, sleep, and cognition in patients with DRE in 6th month after operation to clarify the correlation between sleep and cognition in DRE patients.

**Methods:**

21 individuals with DRE were recruited to enroll in this trial. Each participant completed epileptic focus resection. Seizure frequency was the principle index; the mean seizure frequency was 1 month before surgery and six months after surgery. Cognitive function was assessed by MMSE, and sleep status was assessed by PSQI and ActiGraph; assessments were performed before and 6 months after surgery.

**Results:**

There were significant differences between conditions on all outcome measures; after 6 months of surgery, compared with before treatment, the monthly average seizure frequency of DRE decreased, which was statistically significant (*P* < 0.001) compared with that before treatment. The MMSE score of DRE patients was significantly higher than before (*P* < 0.01), especially the ability of attention, calculation, and recall in MMSE score, which was significantly higher than before operation (respectively, *P* < 0.001 and *P* < 0.01). The subjective sleep evaluation index PSQI and objective measurement of sleep latency, total sleep time, and sleep efficiency of patients with DRE by ActiGraph were statistically significant (respectively, *P* < 0.01) compared with that before treatment. There was a correlation between seizure frequency and MMSE (*r* = −0.8887, *P* < 0.0001), PSQI (0.5515, *P* < 0.01), sleep latency (0.5353, *P* < 0.05), total sleep time (-0.7814, *P* < 0.0001), and sleep efficiency (-0.4380, *P* < 0.05).

**Conclusions:**

Surgery can effectively reduce the epileptic seizures frequency in patients with DRE and indirectly improve the computational power, attention, recall ability, and sleep status of patients. However, this result did not show a correlation between improved cognitive function and sleep, so the patient's cognitive function may be caused by surgery to improve the frequency of seizures. So, whether the improvement of patients' sleep conditions can also significantly improve the frequency of attacks and cognitive function in patients with DRE needs further exploration.

## 1. Introduction

Epilepsy is one of the most common diseases of the nervous system. Epidemiological surveys around the world show that the prevalence of epilepsy is about 7.6% [1]. Despite the variety of treatment options available, approximately, 30–40% of patients with epilepsy still have poor or ineffective antiepileptic drug (AED) treatment and are classified as drug resistant epilepsy (DRE) [2]. The younger the disease, the more likely it is to cause drug-resistant epilepsy [3], especially in patients with childhood-onset; not only the prevalence of DER is high [4]. Furthermore, cognitive dysfunction is present in 64.5% of patients [5, 6]. The link between sleep and epilepsy and cognitive impairment is well established, and different sleep states can affect seizures and interepileptic seizures (IED) [7, 8]. Similarly, epilepsy is associated with an increased incidence of sleep disorders, including insomnia and sleep disruption [9–11]. Sleep disorders can also lead to sleep disruption and deprivation, which can induce further seizures [12]. Neurosurgery is currently the most effective method for treating DRE. Through comprehensive preoperative evaluation and accurate positioning, resection of epileptogenic focus or destruction of epileptic focus is used to eliminate seizures or reduce the frequency or intensity of seizures.

Then, whether the surgical removal of DRE lesions can improve patients' cognitive function and sleep status while improving seizures, we conducted the following research.

## 2. Materials and Methods

### 2.1. Participants

Prior to clinical data collected on 21 DRE patients (age 24.09 ± 3.23 years, duration 11.76 ± 1.87) who underwent surgery from 2015 to 2018, the institution's approval was obtained. The trial was conducted according to the guidelines of the 1964 Helsinki Declaration, and each patient signed written informed consent. The patients originated from inpatients in our hospital. The onset age of patients was 6-16 years old, and the patients were between 18 and 30 years old. DRE-compliant diagnosis (≥4 seizures per month, regular treatment with first-line antiepileptic drugs, and the blood concentration of the drug within the effective range, observation ≥ 2 years) [13] and MMSE score < 24 points, PSQI score > 10 points, and wais − rc score > 70 can cooperate with scale test and instrument inspection. Exclusion criteria for this study are severe cardiopulmonary dysfunction, secondary epilepsy, pregnancy, active psychosis, delirium tremens, and substance abuse with experience of acute withdrawal.

### 2.2. Surgical Treatment

For selected DRE patients, comprehensive clinical manifestations, conventional MRI scan findings, video scalp electroencephalogram (EEG), and neuro electrophysiological manifestations (noninvasive or invasive) are subjected to strict preoperative evaluation and precise positioning; the brain region of epileptogenic area was clearly defined, and a resection scheme was designed for each patient [14, 15].

## 3. Efficacy Evaluation

### 3.1. Primary Evaluation Indicators (Frequency of Seizures)

The number of clinical episodes of epilepsy is a major form of epilepsy, and it is also a major indicator of efficacy. Seizure counts are performed by the patient and/or caregiver [16]. The average monthly frequency of seizures was evaluated 1 month before surgery and 6 months after surgery.

### 3.2. Secondary Evaluation Indicators

Subjects completed two testing sessions: day 7 (prior to surgery) and day 182 (end of the surgery). The evaluation of cognitive function and sleep status was secondary efficacy evaluation, cognitive function is performed using the MMSE, and sleep status is subjectively evaluated by PSQI and objectively evaluated by ActiGraph.

#### 3.2.1. Cognitive Function Evaluation

The Mini-Mental State Examination (MMSE) is used for cognitive screening; the maximum score is 30 points [17, 18]. Cognitive testing included the distribution of orientation, memory, attention and calculation, recall, and language ability.

#### 3.2.2. Subjective Sleep Assessment

The Pittsburgh Sleep Quality Index (PSQI) is a questionnaire used to evaluate the sleep quality, actual sleep, sleep efficiency, sleep disorders, hypnotic drugs, and daytime dysfunction throughout the last month [19]. The total score of PSQI, which falls between 0 and 21, gets the higher the score, the worse the sleep quality.

#### 3.2.3. Objective Sleep Monitoring

According to reports, the ActiGraph (USA/wGT3X-BT, FL 32502) can provide satisfactory objectively measuring of sleep quality [20]. We assessed participants' sleep with ActiGraph. ActiGraph is worn on each participant's nondominant wrist and should not be removed unless it enters the water (such as when bathing or swimming). All participants were tested with ActiGraph for 3 days. Once the measurement is completed, the data is provided with a sleep diary using the ActiLife 6 software (49 E, Chase St, Pensacola, FL 32502, USA), including sleep latency, wake-up times, total sleep time (TST), and sleep efficiency.

## 4. Statistical Analysis

Mean ± standard deviation (Mean ± S) was used to report sample characteristics and outcome measure data. Several paired *t*-tests were completed in order to compare the outcome measures between conditions (presurgery and postsurgery). Possible associations among the quantitative variables were estimated using the Pearson correlation coefficient. All analyses were performed with a significant level of *P* < 0.05, using the statistical pack SPSS 20.0.

## 5. Results

### 5.1. Main Evaluation Indicators (Frequency of Seizures)

Comparing the changes of monthly seizure frequency on the day presurgery and day 182 after surgery, we found that there was significant (*P* < 0.001) difference between presurgery and postsurgery (Figure 1).

### 5.2. Cognitive Function Evaluation

Surgery leads to higher scores of MMSE, calculation, and attention score as well as recall ability score. In Figure 2(a), the score of MMSE in the postsurgery was significantly (*P* < 0.01) higher than that in the presurgery. In Figure 2(b), the score of calculation and attention in the postsurgery was significantly (*P* < 0.01) higher than that in the presurgery (*P* < 0.001). In Figure 2(c), the score of recall ability in the postsurgery was significantly (*P* < 0.01) higher than that in the presurgery (Figures 2(a)–2(c)).

### 5.3. Sleep Status

Surgery reduces PSQI score, shorten sleep latency, and increase total sleep time and sleep efficiency. In Figure 3(a), the score of PSQI in the postsurgery was significantly (*P* < 0.01) lower than in the presurgery. In Figure 3(b), the minutes of sleep latency in the postsurgery were significantly (*P* < 0.01) shorter than that in the presurgery. In Figure 3(c), the total sleep efficiency in the postsurgery was significantly (*P* < 0.01) higher than that in the presurgery. In Figure 3(d), the minutes of total sleep time in the postsurgery were significantly (*P* < 0.01) higher than that in the presurgery (Figures 3(a)–3(d)).

### 5.4. Correlation between Seizure Frequency and Cognitive Function and Sleep Status

Correlation between seizure frequency, cognitive function, and sleep status.  Figure 4: In our analysis of the correlation between seizure frequency, cognitive function, and sleep status. In addition, seizure frequency is strongly correlated with MMSE scores (*r* = −0.8887, *P* < 0.0001), PSQI scores (*r* = 0.5515, *P* < 0.01), sleep latency (*r* = 0.5353, *P* < 0.05), total sleep time (*r* = −0.7814, *P* < 0.0001), and sleep efficiency (*r* = −0.4380, *P* < 0.05) (Figures 4(a)–4(e)).

### 5.5. Correlation between Cognitive Function and Sleep Status

In our analysis of the correlation between cognitive function and sleep status, we found that there was no correlation between MMSE scores and PSQI score (*r* = 0.04285, *P* > 0.05), sleep latency (*r* = 0.08639, *P* > 0.05), total sleep time (*r* = 0.3881, *P* > 0.05), and sleep efficiency (*r* = 0.3880, *P* > 0.05) (Figures 5(a)–5(d)).

### 5.6. Sleep Monitoring by ActiGraph

We adopted objective sleep monitoring by ActiGraph for 3 days of pre- and postsurgery, to observe the change of sleep latency, total sleep time, and sleep efficiency. It was found that the sleep latency shorted, total sleep time lengthened, and sleep efficiency improved after surgery (Figure 6).

## 6. Discussion

Epilepsy is a brain disease that is caused by abnormal simultaneous firing of brain neurons and is characterized by transient central nervous system dysfunction. So far, although there are more than 20 antiepileptic drugs (AED), one-third of patients still have poor clinical treatment and become DRE [21]. DRE often recurs, which not only seriously affects patients' quality of life, causes patients with cognitive dysfunction, psychological and emotional problems, and sleep disorders but also bring a heavy economic burden on the family and society. Under the premise that scientific and reasonable screening meets the standards of surgery, surgery is currently considered to be an effective treatment for DRE [22, 23]. A clinical study of the frequency of postoperative seizures and psychological evaluation for up to 15 years in patients with DRE showed that 32% of patients had no seizures and 75% of patients had a good prognosis [24]. The effect of surgical treatment should not only evaluate the changes in the frequency and form of seizures of the patients after surgery but also include the cognitive function, sleep status, psychology, and emotions of patients after the surgical treatment in the evaluation of surgical efficacy [25]. Cognitive dysfunction is a common accompanying symptom in patients with epilepsy, and cognitive dysfunction exists in 64.5% of children with epilepsy, mainly due to decreased attention, memory, judgment, and other aspects [6]. In general, the younger the age of onset of epilepsy, the more severe the cognitive impairment [26]; while epilepsy is closely related to sleep, seizures themselves cause sleep disorders such as reduced total sleep time and prolonged sleep latency [27] may cause epileptic discharge or seizures [28].

In this study, 21 cases of DRE patients with sleep problems and cognitive dysfunction admitted to our hospital were given surgical treatment. The results showed that the monthly frequency of epilepsy was significantly lower than that before treatment at 6 months after treatment (*P* < 001); further research results show that the MMSE score is statistically significant compared with the preoperative comparison (*P* < 0.001), of which the attention and calculation ability and recall ability are statistically significant compared with the preoperative difference (respectively, *P* < 0.0001 and *P* < 0.001), indicating that surgical treatment of DRE has a better effect on patients' attention and computing power and recall ability. In this study, the PSQI of DRE patients after treatment was significantly improved compared with that before treatment (*P* < 0.01). Whether in sleep latency, total sleep time, or sleep efficiency, it was significantly improved compared with before treatment (*P* < 0.01). It shows that while surgical treatment of DRE can improve seizures, it can also improve patient's sleep. Correlation analysis of postoperative seizures with cognitive ability and sleep therapy in patients with DRE found that the frequency of seizures was strongly correlated with MMSE score, PSQI score, sleep latency, total sleep time, and sleep efficiency (*P* < 0.0001, *P* < 0.01, *P* < 0.05, *P* < 0.0001, *P* < 0.05). However, the MMSE scores of patients with DRE did not show any correlation with PSQI score, sleep latency, total sleep time, and sleep efficiency (*P* > 0.05). This shows that surgery can improve the frequency of seizures, improve cognitive function and sleep therapy in patients with DRE, and has positive clinical application value. Surgery improves the attention, calculation, and recall ability of patients with DRE, as well as the sleep latency, total sleep time, and sleep efficiency of patients. However, there is no correlation between sleep improvement in DRE patients and changes in cognitive level. Perhaps the frequency of attacks in DRE patients is the cause of cognitive impairment.

## 7. Conclusions

In summary, surgery can effectively control the frequency of seizures in patients with DRE, thereby improving patients' cognitive function and sleep quality. However, whether the clinical improvement of sleep quality in DRE patients and whether they can agree to reduce the frequency of seizures and improve cognitive function in DRE patients remain to be analyzed in the future.

## Figures and Tables

**Figure 1:** Analysis of the impact of surgery on monthly seizure frequency in DRE patients. Note: Compared with presurgery, ^∗∗^*P* < 0.01, ^∗∗∗^*P* < 0.001. 1: main evaluation indicators (frequency of seizures). Comparing the changes of monthly seizure frequency on the day presurgery and day 182 after surgery, we found that there was significant difference between presurgery and postsurgery (*P* < 0.001).

**Figure 2:** Surgery leads to higher scores of MMSE, calculation, and attention score as well as recall ability score. In (a), the score of MMSE in the postsurgery was significantly higher than that in the presurgery (*P* < 0.01). In (b), the score of calculation and attention in the postsurgery was significantly higher than that in the presurgery (*P* < 0.001). In (c), the score of recall ability in the postsurgery was significantly higher than that in the presurgery (*P* < 0.01).

**Figure 3:** Surgery reduces PSQI score, shorten sleep latency, and increase total sleep time and sleep efficiency. (a) The score of PSQI in the postsurgery was significantly lower than in the presurgery (*P* < 0.01). (b) The minutes of sleep latency in the postsurgery were significantly shorter than that in the presurgery (*P* < 0.001). (c) The total sleep efficiency in the postsurgery was significantly higher than that in the presurgery (*P* < 0.01). (d) The minutes of total sleep time in the postsurgery were significantly higher than that in the presurgery (*P* < 0.01).

**Figure 4:** Correlation between seizure frequency, cognitive function, and sleep status. In our analysis of the correlation between seizure frequency, cognitive function, and sleep status. In addition, seizure frequency is strongly correlated with MMSE scores (*r* = −0.8887, *P* < 0.0001), PSQI scores (*r* = 0.5515, *P* < 0.01), sleep latency (*r* = 0.5353, *P* < 0.05), total sleep time (*r* = −0.7814, *P* < 0.0001), and sleep efficiency (*r* = −0.4380, *P* < 0.05) (a–e).

**Figure 5:** Correlation between cognitive function and sleep status. In our analysis of the correlation between cognitive function and sleep status, we found that there was no correlation between MMSE scores and PSQI score (*r* = 0.04285, *P* > 0.05), sleep latency (*r* = 0.08639, *P* > 0.05), total sleep time (*r* = 0.3881, *P* > 0.05), and sleep efficiency (*r* = 0.3880, *P* > 0.05) (a–d).

**Figure 6:** 3 days' objective sleep monitoring by ActiGraph.

## Data Availability

The datasets used and/or analyzed during the current study are available from the corresponding author on reasonable request.
